# Short-Term Load Forecasting Based on EEMD-WOA-LSTM Combination Model

**DOI:** 10.1155/2022/2166082

**Published:** 2022-08-24

**Authors:** Lei Shao, Quanjie Guo, Chao Li, Ji Li, Huilong Yan

**Affiliations:** ^1^School of Electrical Engineering and Automation, Tianjin University of Technology, Tianjin 300384, China; ^2^School of Precision Instrument and Opto-Electronics Engineering, Tianjin University, Tianjin 300384, China

## Abstract

The purpose of this study was to better apply artificial intelligence algorithm to load forecasting and effectively improve the forecasting accuracy. Based on the long short-term memory neural networks, a combined model based on whale bionic optimization is proposed for short-term load forecasting. The whale bionic algorithm is used to solve the problem that the long short-term memory neural networks are easy to fall into local optimization and improve the accuracy of parameter optimization. The original signal is decomposed into multiple characteristic components by set empirical mode decomposition. Each feature component is input into the bionic optimized combination model for prediction. Finally, get the load forecasting results. Compared with the prediction results of EEMD-ARMA model, RNN model, LSTM model, and WOA-LSTM model, the combined prediction model optimized by whale bionics has less prediction error and higher prediction accuracy.

## 1. Introduction

Due to the intelligence and progressiveness of artificial intelligence technology, artificial intelligence technology has been applied in aerospace, medical and health, power system, and many other fields. The application of artificial intelligence technology in power system and power enterprises can optimize the stability and security of power system. Due to the increasing complexity of power system load, power load forecasting has become a key technology for the stable operation of the system. The development of short-term load forecasting has also changed from basic mathematical methods to artificial intelligence forecasting. The prediction accuracy is improved by combining artificial intelligence algorithm.

There are three kinds of short-term power load forecasting methods: traditional forecasting method, modern forecasting method, and combined forecasting model method. Traditional prediction methods include regression prediction method [1], exponential smoothing method, [2], and time series method [3]. The prediction accuracy of regression prediction method is low, but the fitting speed is fast. It is a basic prediction model. Exponential smoothing method can get the contribution of all data to the prediction data through different weights. Exponential smoothing method has poor ability to judge the turning point of data. The advantage of time series method is that it can eliminate random fluctuations. The disadvantage is that the time series method is greatly affected by the original data, and the fitting accuracy is poor when the amount of data is large.

Modern prediction methods include grey prediction method, fuzzy prediction method, and neural network method. Jin et al. [4] proposed a new grey relational competition model for short-term power load forecasting. When the amount of data of load series increases and the degree of dispersion increases, the prediction accuracy of grey prediction method will decrease. Cevik and Cunkas [5] proposed a short-term load forecasting model based on fuzzy logic and adaptive neuro fuzzy inference system (ANFIS). The fuzzy control algorithm based on fuzzy logic and fuzzy mathematics in fuzzy theory is often used in the field of power load. However, this method has high dependence on experience, poor adaptive learning ability, and poor prediction effect on nonlinear data. Neural networks (NNs) are the most widely used prediction methods [6–8], and build a multifunctional computing model. In neural network model, radial basis function and error back propagation algorithm are widely used. Various neural network structures have been proposed to improve the prediction effect [9–11]. With the rapid development of artificial intelligence, many experts and scholars have proposed deep neural network. Compared with traditional neural network, deep neural network (DNN) [12] has multiple hidden layers, which enhances the sensitivity to the correlation of temporal data.

Typical deep neural networks include convolutional neural network (CNN), deep confidence network, and recurrent neural network (RNN). RNN is proposed to better process sequence information [13]. LSTM evolved from RNN [14] and was first developed by Hochreiter [15], which solves the problems of gradient disappearance and gradient explosion that are easy to occur in RNN and can retain short-term and long-term memory in the network [16]. LSTM has also been successfully applied in many research fields [17], such as phoneme classification [18], traffic prediction [19], language subtitles [20], and action recognition [21]. LSTM can effectively learn the law information in the historical sequence information. In the above research fields, LSTM model has achieved high accuracy, and it is a very efficient neural network model.

A single neural network prediction algorithm is easy to fall into local optimization during testing. The complexity of power load also leads to the fact that a single prediction method cannot ensure the accuracy of prediction. Combined prediction model is proposed to solve the problem of prediction accuracy. The combination of different types of artificial neural network models is a research hotspot to solve the problem of short-term power load forecasting. Santra and Lin [22] proposed a combined model of genetic algorithm (GA) and long-term and short-term memory (LSTM). GA is used to optimize the parameters of LSTM to improve the robustness of short-term load forecasting. However, at present, the selection of parameters of genetic algorithm mostly depends on experience, such as crossover rate and mutation rate. And the genetic algorithm is slow to deal with the feedback information of the network, and the search speed of the algorithm is slow. Hong et al. [23] proposed a short-term load forecasting model based on deep neural network and iterative ResBlock to learn the correlation between different power consumption behaviors. Compared with the traditional convolutional neural network, iterative ResBlock can transmit low-level information and make the network training deeper. But the deeper network structure needs better GPU to train, and the requirements for hardware are higher. Moradzadeh et al. [24] proposed a combined model of improved support vector regression (SVR) and long-term and short-term memory (LSTM), which achieved good prediction results. However, support vector regression is not suitable for large data sets. When the number of features of each data point exceeds the number of training data samples, support vector regression performs poorly. And when the data set is noisy, it is easy to cause the target classes to overlap. He et al. [25] proposed a combined prediction model based on variational modal decomposition and long-term and short-term memory networks. The original input signal is processed by variational modal decomposition, which reduces the interference of noise. However, the parameter selection of LSTM will affect the prediction accuracy of the whole combined model. Meng et al. [26] proposed a long-term and short-term memory neural network model combining empirical mode decomposition and attention mechanism. The performance of LSTM neural network is optimized. However, empirical mode decomposition (EMD) has a serious mode aliasing phenomenon, which requires high requirements for the original data. Set empirical mode decomposition (EEMD) is proposed to solve the mode aliasing phenomenon in EMD.

To sum up, consider the raw data processing and parameter selection. The set empirical mode decomposition is used to process the original signal to overcome the phenomenon of modal aliasing. The whale bionic optimization algorithm is used to optimize the parameters. In this paper, we propose an LSTM neural network model optimized by whale bionic algorithm for short-term load forecasting. The model combines bionic algorithm with artificial intelligence algorithm. The data is decomposed into modal components of different scales as the input of the model through set empirical mode decomposition. WOA layer optimizes LSTM parameters according to whale algorithm. The LSTM layer is used to model historical data. Based on the historical load data of a company, the artificial intelligence method is evaluated. Compared with RNN model, LSTM model, EEMD-ARMA model, and WOA-LSTM model, the proposed prediction method has higher accuracy.

The remainder of this article is summarized as follows. The second section introduces the basic principles of LSTM neural network, whale algorithm, and EEMD. The third section introduces the combined forecasting model and error evaluation index. The fourth section gives the relevant example analysis. The fifth section makes a summary.

## 2. Algorithm Preparation

### 2.1. LSTM

When ordinary recurrent neural network (RNN) processes complex data, improper parameter selection is easy to lead to gradient disappearance and gradient explosion. Compared with RNN, LSTM neural network adds logic gate control mechanism and state transfer unit, so that it not only retains the correlation with time but also increases the dependence between distant information.  Figure 1 shows the cell unit of LSTM neural network. *x*_*t*_ in the figure is the input data at time *t*. *h*_*t*−1_ is the output of the hidden layer at time *t* − 1. *c*_*t*−1_ is the state of cell unit at time *t* − 1. *c*_*t*_ is the state of cell unit at time *t*. *σ* represents the sigmoid function. Output value *h*_*t*_ of LSTM neural network and unit status *c*_*t*_ at the current time are determined by the input value *x*_*t*_ at the current time and output value of hidden layer at last time *h*_*t*−1_ and unit status *c*_*t*−1_ shared decision.

The calculation formula is

(1) $$\begin{array}{c} f_{t}=\sigma \left(W_{f}\cdot \left[h_{t-1},x_{t}\right]+b_{f}\right), \end{array}$$

(2) $$\begin{array}{c} i_{t}=\sigma \left(W_{i}\cdot \left[h_{t-1},x_{t}\right]+b_{i}\right), \end{array}$$

(3) $$\begin{array}{c} {\tilde{c}}_{t}=\tanh\left(W_{c}\cdot \left[h_{t-1},x_{t}\right]+b_{c}\right), \end{array}$$

(4) $$\begin{array}{c} c_{t}=f_{t}*c_{t-1}+i_{t}*{\tilde{c}}_{t}, \end{array}$$

(5) $$\begin{array}{c} h_{t}=\sigma \left(W_{o}\left[h_{t-1},x_{t}\right]+b_{o}\right)*\tanh\left(c_{t}\right). \end{array}$$

In the formula, *f*_*t*_, *i*_*t*_, ${\tilde{c}}_{t}$, *c*_*t*_, and *h*_*t*_are forgetting gate, input gate, input node, cell state, and output layer, *W*_*f*_, *W*_*i*_, *W*_*c*_, *W*_*o*_ and *b*_*f*_, *b*_*i*_, *b*_*c*_, *b*_*o*_ is the weight matrix of forgetting gate, *b*_*f*_ is the weight matrix and offset term corresponding to forgetting gate, input gate, input node, and output gate, and *σ* is the sigmoid function.

### 2.2. Whale Optimization Algorithm

Bionic intelligent algorithms have developed rapidly, such as particle swarm optimization, leapfrog algorithm, and fish swarm algorithm. Mirjalili and Lewis creatively put forward whale optimization algorithm in the field of bionic intelligent algorithm [27]. Compared with other algorithms, whale algorithm is an intelligent optimization algorithm with simple operation, few parameters, and good optimization performance. By simulating the whale predation mechanism to represent the optimization process of the algorithm, the global and local search capabilities are better weighed and quantified. The flow chart is shown in Figure 2.

In WOA, search particles are initialized in space. When |*A*| < 1, WOA enters local search; when |*A*| > 1, WOA enters the global search. The formula is as follows:

(6) $$\begin{array}{c} a\left(t\right)=2-\frac{2t}{T}, \end{array}$$

(7) $$\begin{array}{c} A\left(t\right)=2a\left(t\right)r-a\left(t\right), \end{array}$$

(8) $$\begin{array}{c} C\left(t\right)=2r. \end{array}$$

In the formula, *t* represents the current number of iterations and *T* represents the maximum number of iterations. *r* is any value between [0, 1]. In the whole iterative process, *a* gradually decreases from 2 to 0. *A* is a random number belonging to [−*a*, *a*].

WOA enters the local search phase. One is the shrink surrounding method and the other is the spiral update method. The formula for the contraction phase is as follows:

(9) $$\begin{array}{c} \overset{⟶}{X}\left(t+1\right)=\overset{⟶}{X^{*}}\left(t\right)-A\left(t\right)\cdot \overset{⟶}{D}\left(t\right), \end{array}$$

(10) $$\begin{array}{c} \overset{⟶}{D}\left(t\right)=\left|C\left(t\right)\cdot \overset{⟶}{X^{*}}\left(t\right)-\overset{⟶}{X}\left(t\right)\right|. \end{array}$$

$\overset{⟶}{D}$ stands for random distance, which is the distance between the target and the search particle. The spiral update method formula is as follows:

(11) $$\begin{array}{c} \overset{⟶}{X}\left(t+1\right)=\overset{⟶}{D^{\prime }}\left(t\right)\cdot e^{bl}\cdot \cos\left(2\pi l\right)+\overset{⟶}{X^{*}}\left(t\right), \end{array}$$

(12) $$\begin{array}{c} \overset{⟶}{D^{\prime }}\left(t\right)=\left|{\overset{⟶}{X}}^{*}\left(t\right)-\overset{⟶}{X}\left(t\right)\right|. \end{array}$$

*X* ^∗^ represents the optimal solution so far. $\overset{⟶}{D}$ represents the random distance between the target prey and the search particle. $\overset{⟶}{D^{\prime }}$ represents the distance between the optimal solution and the search particle, *b* is a constant coefficient, and *l* is a random number in [-1,1]. *p* is a probability randomly generated from [0,1].

When |*A*| > 1, WOA enters the global search phase. The formula is as follows:

(13) $$\begin{array}{c} \overset{⟶}{X}\left(t+1\right)=\overset{⟶}{X_{\mathrm{rand}}}-A\left(t\right)\cdot \overset{⟶}{D}\left(t\right), \end{array}$$

(14) $$\begin{array}{c} \overset{⟶}{D}\left(t\right)=\left|C\left(t\right)\cdot \overset{⟶}{X_{\mathrm{rand}}}-\overset{⟶}{X}\left(t\right)\right|. \end{array}$$

$\overset{⟶}{X_{\mathrm{rand}}}$ represents the search particles randomly selected from the population.

The optimization process of whale optimization algorithm is as follows:

1. Initialize the whale population
2. In the process of evolution, whales update their position according to the optimum
3. Determine the whale position update method according to *p*
4. Iterate until the whale algorithm meets the termination requirements

The whale algorithm is used to optimize the parameters of LSTM model. In this paper, MAPE is used as the loss function of whale algorithm. When the loss value meets the requirements, the optimized parameter value is obtained. The definition formula of fitness function Training Loss is as follows:

(15) $$\begin{array}{c} \text{Training Loss}=\text{MAPE}\left(h,y\right)=\frac{1}{n}\overset{n}{\underset{i=1}{\sum }}\left|\frac{h\left(i\right)-y\left(i\right)}{y\left(i\right)}\right|. \end{array}$$

*h*(*i*) is the *i*th predicted value in the predicted results, *y*(*i*) is the *i*th true value in the data samples, and *n* is the number of predicted samples. The more accurate the forecast value is, the smaller the loss value will be.

The detailed process is as follows:

1. Initialization of LSTM model parameters
2. Whale algorithm population initialization. A set of values composed of these three variables (*n*, *ε*, iter) are input into the whale algorithm as parameters to be optimized. The three parameters represent the number of hidden layer nodes, learning rate, and iteration times, respectively
3. Take the initialized value as the historical optimal value to assign and train the parameters of LSTM
4. Set the Training Loss obtained from the traditional LSTM training as the system requirement, and calculate the model loss value optimized by the whale algorithm
5. If the loss value of the model optimized by whale algorithm is less than Training Loss, the requirements are met, and the final prediction model and parameter values are output
6. If the loss value cannot be less than Training Loss or the number of iterations does not reach the maximum, update the parameters and retrain. Otherwise, stop training

### 2.3. Ensemble Empirical Mode Decomposition

When dealing with time series problems, EMD decomposition can stabilize the data. EMD can decompose the nonlinear and nonstationary signal into a series of IMF components, which are the local characteristic signals of different scales of the original signal.

Mode aliasing may occur in EEM mode decomposition. EEMD will add Gaussian white noise before decomposition and then EMD decomposition. In order to minimize the influence of white noise on the original sequence, repeat the experiment for many times, and finally, calculate the mean value of multiple groups of results. The decomposition steps of EEMD are as follows:

1. Set the number of decomposition *m*
2. The Gaussian white noise is added to the original sequence *x* (*T*). The standard deviation of the added white noise is usually 0.2 times of the standard deviation of the original sequence, and the mean value is 0. The sequence formula after adding white noise is obtained as follows:

(16) $$\begin{array}{c} x^{\prime }\left(t\right)=x\left(t\right)+\varepsilon^{n}\left(t\right). \end{array}$$

In the formula *ε*^*n*^(*t*)(*n* = 1, 2, ⋯, *m*) is random Gaussian white noise, and *m* is the length of the original sequence

(3) After the previous step, we obtained all the *IMF*_*i*_^*n*^(*t*)(*n* = 1, 2, ⋯, *m*); *i* is the order of IMF
(4) Repeat steps 2 and 3 *m* times to get all IMF
(5) The noise interference can be eliminated by averaging the *m* times of IMF. The formula is as follows:

(17) $$\begin{array}{c} \overset{¯}{\text{IM}{\text{F}}_{i}}=\frac{1}{m}\overset{m}{\underset{n=1}{\sum }}\text{I}\text{M}{\text{F}}_{i} \end{array}$$

Unlike EMD, EEMD results are not necessarily the same. It varies with the magnitude of white noise, so the EEMD decomposition cannot obtain a unique solution. Even if the same parameters are selected, the calculated results are still different due to the randomness of the noise. However, as the number of tests increases, the influence can be offset when calculating the mean value. As long as the number of tests is enough, the results will tend to be consistent. In addition to the influence of the magnitude of Gaussian white noise on the decomposition results, the percentage also has a great influence on the results. If the percentage is too small, the effect is small or not. If the percentage is too large, it will cause interference and large error. At present, the more effective method to reduce interference is to have enough average times. Generally, when the average times is hundreds of times, the effect is good.

## 3. Main Result

### 3.1. EEMD-WOA-LSTM Combined Model

Figure 3 shows the framework of the model proposed in this paper. The EEMD-WOA-LSTM method proposed in this paper includes three stages: data decomposition, component prediction, and prediction result reconstruction.

EEMD-WOA-LSTM model makes full use of EEMD's ability to avoid component mode aliasing and WOA-LSTM's long-term memory of data. The three stages are as follows:

1. EEMD performs data decomposition. Output multiple modal components with different characteristics
2. Each IMF subsequence is predicted separately. For each component, an LSTM network is established to study its internal dynamic change law. Use WOA algorithm to update the LSTM network
3. Normalize the prediction results of each IMF subsequence and superimpose the prediction values of each component

### 3.2. Prediction and Evaluation Index

In this paper, several commonly used error evaluation indexes in power load forecasting are adopted: mean absolute error (MAE), root mean square error (RMSE), and mean absolute percent error (MAPE).

1. Mean absolute error (MAE):

(18) $$\begin{array}{c} \text{MAE}\left(h,y\right)=\frac{1}{n}\overset{n}{\underset{i=1}{\sum }}\left|h\left(i\right)-y\left(i\right)\right| \end{array}$$

(2) Root mean square error (RMSE):

(19) $$\begin{array}{c} \text{RMSE}\left(h,y\right)=\sqrt{\frac{1}{n}\overset{n}{\underset{i=1}{\sum }}{\left(h\left(i\right)-y\left(i\right)\right)}^{2}} \end{array}$$

(3) Mean absolute percentage error (MAPE):

(20) $$\begin{array}{c} MAPE\left(h,y\right)=\frac{1}{n}\overset{n}{\underset{i=1}{\sum }}\left|\frac{h\left(i\right)-y\left(i\right)}{y\left(i\right)}\right| \end{array}$$

In the formula, *h*(*i*) is the *i*th predicted value in the prediction result, *y*(*i*) is the ith true value in the data sample, and *n* is the number of prediction samples.

### 3.3. LSTM Prediction Accuracy Analysis

Select the load data of one equipment in the factory from April 1, 2018, to May 30, 2018, one sampling point at the same time every day, a total of 60 load data, as shown in Figure 4.

During this period, the production plan of this equipment is almost the same. The plant has constant temperature and humidity throughout the year, so the power consumption is not affected by the external environment, and the data fluctuation is small. Take the raw data of the next 15 days as the test set. Through the simulation of RNN and LSTM prediction models, it is verified that LSTM has better prediction effect than RNN model. The number of hidden layer nodes of neural network is set as 18, the learning rate is 0.002, and the number of iterations is 200.

The 15-day power load forecasting results of RNN and LSTM models are shown in Figures 5 and 6, respectively.

Calculate the regression evaluation index according to equations (18)-(20), and get the MAE, RMSE, and MAPE of the two algorithms, as shown in Table 1.

As a whole, the prediction result of LSTM model is closer to the real curve, while the prediction result of RNN model deviates greatly. And the three evaluation indexes of LSTM model in Table 1 are smaller than those of RNN model.

At present, the method to determine the number of nodes in the hidden layer depends on experiments. Generally, some representative nodes are selected for simulation, and the interval of the optimal solution is determined through the simulation results, and the experiment is continued. Select the optimal number of hidden layer nodes as the final result. Fix other parameters unchanged, select some representative hidden layer nodes, and get the prediction result curve as shown in Figure 7. The error values of each prediction result are shown in Table 2.

The results in Table 2 show that the prediction results vary with the number of hidden layer nodes. When the number of hidden layer nodes is less than 10, the three indicators are larger and the prediction accuracy is lower. When it is 10, the prediction accuracy increases significantly, and when the number of hidden layer nodes is more than 20, the accuracy decreases.

The advantages of the LSTM algorithm are as follows:

1. LSTM has better fitting effect in processing complex data
2. LSTM solves the problem of dependence on memory or forgetting for such information that is far away from each other
3. In the prediction comparison of the above two models, it is found that the MAE, RMSE, and MAPE of RNN are 12.048, 12.806, and 0.939, respectively, and the MAE, RMSE, and MAPE of LSTM neural network are 8.556, 9.576, and 0.665, respectively, which improves the accuracy by 29.0%, 25.2%, and 29.2%, respectively. Compared with various error evaluation indicators, LSTM model has better prediction results and can be used as a good model in the field of power load forecasting

### 3.4. Combined Forecast Model Data

In this paper, the real load data of a factory from January 1, 2019, to December 31, 2020, is taken as the original data. The sampling interval is 24 hours, that is, one sampling point per day. The original data curve is shown in Figure 8. Through the training of the data, predict the power consumption data in the next 30 days. In this paper, RNN model, LSTM model, EEMD-ARMA model, WOA-LSTM model, and EEMD-WOA-LSTM model are used for prediction and data analysis.

### 3.5. Decomposition of Original Load Series

EMD and EEMD were used to decompose the time series of the plant. The comparison of EMD and EEMD decomposition data is shown in Figures 9 and 10.

IMF9 in Figure 9 and IMF9 in Figure 10 are respective trend items. In Figure 9, mode aliasing occurs. It can be seen from Figure 10 that EEMD overcomes the problem of modal aliasing and can decompose the power load signal into different frequencies with distinct characteristics. In order to achieve better prediction accuracy. We use EEMD for data decomposition. The decomposed feature components are input into the prediction model for learning.

### 3.6. Analysis of Experimental Results

In this paper, the rolling prediction method is used for model training, and RNN and LSTM prediction models are established for analysis. The number of hidden layer nodes of neural network is set as 80, the learning rate is 0.01, and the number of iterations is 500.

The prediction results of RNN model are shown in Figure 11. The results predicted by RNN are intuitively more accurate than the traditional algorithm. However, for the extreme points, the RNN algorithm has poor fitting degree and the result deviation is large.

The LSTM model is used to predict the data. The prediction results are shown in Figure 12. From the visual point of view, the prediction results by LSTM neural network have improved the accuracy. The prediction for the data with small change range is relatively accurate. However, because the parameters are difficult to determine, the results have a certain offset for the data near the extreme points, and the overall prediction accuracy is not too high.

The number of components generated by EEMD decomposition depends on how many ARMA models need to be established, and each ARMA model is also different. In fact, the data samples decomposed by EEMD meet the requirements of ARMA modeling, that is to say, they are all stable sequences. Therefore, the process of stability determination is omitted. Generally, AIC and BIC are used to determine the order. However, when selecting the order, there is a large amount of calculation, so the well-known ergodic method is usually used. So fixed order modeling is a good method, and this paper adopts this method. The first step in the EEMD-ARMA data prediction process is to use EEMD to decompose the data, then model each component separately for training, and finally superimpose the prediction results. The prediction curve is shown in Figure 13.

The WOA-LSTM model was used for analysis. Due to the large amount of data, the initial population size of whale algorithm is 50, the initial iteration times is 500, and the initialization parameters (*n*, *ε*, iter) are [10,100], [0.001,0.01], and [400,1000]. Through the optimization of LSTM neural network by WOA, the obtained combined model can better optimize the parameters of LSTM. It can better predict and fit the whole or at the peak, trough, and inflection point of extreme points than the previous algorithms, and the prediction accuracy is significantly improved. The prediction results are shown in Figure 14.

Finally, the EEMD-WOA-LSTM model is used to analyze and predict the load data. The prediction results are shown in Figure 15. Compared with WOA-LSTM model, this model has more accurate prediction results, higher fitting degree with real data, and higher prediction accuracy.

## 4. Results

The comparison of prediction results of the five models is shown in Figure 16. Calculate the regression evaluation indexes according to formula (18)-(20), and get three error evaluation indexes of the five models, as shown in Table 3. The prediction results of each model are shown in Table 4.

For RNN model, LSTM model, and WOA-LSTM model, the coincidence degree between the predicted value and the real value curve of the obtained results from high to low is WOA-LSTM model, LSTM model, and RNN model. WOA-LSTM model is the closest training model to real data samples among the three, which shows that LSTM neural network optimized by whale optimization algorithm has good training effect for large and small-scale data training samples.

For all models, in the part where the real curve fluctuates little, the fitting degree of several algorithms is good, but at the extreme point, the fitting degree of EEMD-ARMA and LSTM models is poor. Although the original LSTM model is better than EEMD-ARMA model on the whole, there is a certain gap between the extreme point and the real value. The optimized WOA-LSTM model can fit the real curve well both in the whole and at the extreme points. EEMD-WOA-LSTM model has better prediction effect, and the fitting degree with the original data is the highest among these models. Compared with the WOA-LSTM model, the MAE of EEMD-WOA-LSTM model decreased by 30.6%, RMSE decreased by 35.1%, and MAPE decreased by 29.6%.

## 5. Discussion

This paper combines bionic algorithm and artificial intelligence algorithm and proposes an EEMD-WOA-LSTM combined model. EEMD is used to decompose the original load series into multiple characteristic components. The neural network is optimized by the whale algorithm and used to predict each component. The components obtained from the prediction are superimposed to form the final prediction result. The method is applied to the power load forecasting of a factory. The simulation results show that, compared with other methods listed in the paper, the EEMD-WOA-LSTM model has the lowest prediction error of 0.019 (MAPE) and high prediction accuracy. It is an ideal short-term load forecasting model. The artificial intelligence algorithm can be well applied to load forecasting to achieve efficient and accurate short-term load forecasting.

## Figures and Tables

**Figure 1:** LSTM neural network unit.

**Figure 2:** Flow chart of whale optimization algorithm.

**Figure 3:** EEMD-WOA-LSTM model framework.

**Figure 4:** Raw data.

**Figure 5:** Comparison of RNN prediction results.

**Figure 6:** Comparison of LSTM prediction results.

**Figure 7:** Prediction results of nodes in different hidden layers.

**Figure 8:** Raw data curve.

**Figure 9:** EMD decomposition data curve.

**Figure 10:** EEMD decomposition data curve.

**Figure 11:** RNN data comparison chart.

**Figure 12:** LSTM data comparison chart.

**Figure 13:** EEMD-ARMA data comparison chart.

**Figure 14:** WOA-LSTM data comparison chart.

**Figure 15:** EEMD-WOA-LSTM data comparison chart.

**Figure 16:** Comparison of prediction data of five models.

**Table 1:** Calculation results of evaluation indicators of two algorithms.

Algorithm type	MAE	RMSE	MAPE
RNN	12.048	12.806	0.939
LSTM	8.556	9.576	0.665

**Table 2:** Prediction error of nodes in different hidden layers.

Hidden layer nodes	MAE	RMSE	MAPE
5	9.280	11.238	0.720
10	9.117	11.107	0.703
20	11.155	13.395	0.865
30	12.809	15.116	0.995
40	11.265	13.623	0.874

**Table 3:** Calculation results of regression evaluation indexes of prediction model.

Algorithm type	MAE	RMSE	MAPE
EEMD-ARMA	25.884	35.723	0.083
RNN	24.581	33.011	0.079
LSTM	12.113	15.254	0.039
WOA-LSTM	8.376	10.773	0.027
EEMD-WOA-LSTM	5.812	6.989	0.019

**Table 4:** Prediction results of each model.

Sample point	Real data	EEMD-ARMA	RNN	LSTM	WOA-LSTM	EEMD-WOA-LSTM
1	31255.53	31261.36	31265.21	31263.57	31259.36	31253.06
2	31213.88	31267.36	31266.36	31220.99	31210.03	31215.70
3	31245.61	31237.54	31230.25	31238.15	31240.52	31242.01
4	31253.90	31262.31	31243.36	31245.07	31258.33	31255.05
5	31220.98	31265.14	31255.51	31262.04	31246.29	31217.46
6	31263.84	31248.10	31245.36	31245.27	31260.36	31265.36
7	31263.86	31278.23	31250.31	31260.73	31270.58	31266.14
8	31172.79	31280.32	31255.36	31210.84	31190.64	31175.63
9	31248.67	31229.36	31230.31	31239.17	31243.35	31244.65
10	31263.06	31270.56	31275.31	31262.67	31260.25	31267.99
11	31262.59	31283.65	31280.36	31276.22	31268.47	31276.58
12	31263.84	31280.16	31248.36	31254.66	31260.36	31268.73
13	31230.94	31220.66	31250.32	31221.76	31225.74	31226.41
14	31166.04	31223.36	31208.04	31157.22	31177.51	31179.76
15	31124.32	31190.21	31192.34	31149.26	31148.15	31133.88
16	31261.80	31272.38	31210.24	31252.24	31250.85	31256.07
17	31271.93	31300.21	31284.14	31277.48	31280.69	31276.20
18	31288.68	31302.32	31278.34	31298.77	31293.64	31284.17
19	31251.52	31260.12	31236.65	31246.78	31257.12	31247.55
20	31213.71	31230.37	31225.21	31222.19	31221.25	31225.95
21	31250.40	31238.21	31238.64	31241.57	31244.55	31252.89
22	31242.72	31250.14	31231.21	31234.73	31240.89	31247.52
23	31251.60	31230.21	31262.35	31237.27	31245.64	31246.98
24	31243.60	31250.39	31234.36	31240.71	31244.62	31244.58
25	31310.12	31240.14	31223.42	31281.82	31300.66	31303.91
26	31204.21	31270.25	31215.32	31214.91	31231.64	31211.85
27	31262.06	31240.18	31253.36	31248.29	31252.36	31250.82
28	31235.40	31253.21	31242.31	31247.48	31240.25	31248.36
29	31269.14	31260.99	31230.32	31258.01	31254.36	31257.52
30	31214.37	31226.34	31225.36	31207.32	31210.31	31220.65

## Data Availability

The load forecasting data used to support the results of this study has not been provided because it is private data of enterprises.
